# Deep Learning Model for the Image Fusion and Accurate Classification of Remote Sensing Images

**DOI:** 10.1155/2022/2668567

**Published:** 2022-11-22

**Authors:** S. Roselin Mary, Sunita Pachar, Prabhat Kumar Srivastava, Medhavi Malik, Avani Sharma, Tariq G. Almutiri, Zabihullah Atal

**Affiliations:** ^1^Department of CSE, Anand Institute of Higher Technology, Kalasalingam Nagar, Kazhipattur, OMR, Chennai 603103, India; ^2^President Vasundhara Blessing Foundation, Academician GLA University, Chaumuhan, India; ^3^Computer Science and Engineering Department, IMS Engineering College, Ghaziabad, UP, India; ^4^School of Computing Science and Engineering, Galgotias University, Noida, India; ^5^Department of Information Technology, Manipal University Jaipur, Jaipur, India; ^6^Department of Computer Science, Community College, King Saud University, Riyadh 11437, Saudi Arabia; ^7^Department of Computer Science, Faculty of Computer Science, Kardan University, Afghanistan

## Abstract

Deep learning is widely used for the classification of images that have various attributes. Image data are used to extract colour, texture, form, and local features. These features are combined in feature-level image fusion to create a merged remote sensing image. A trained depth belief network (DBN) processes and divides fusion images, while a Softmax classifier determines the land type. As tested, the proposed approach can categorise all types of land. Traditional methods of detecting distant sensing photographs have limitations that can be overcome by using convolutional neural networks (CNN). Traditional techniques are incapable of combining deep learning elements while doing badly in classification. After PCA decreases data dimensionality, deep learning is applied to generate effective features that employ deep learning after PCA has reduced the dimensionality of the data. Principal component analysis is commonly used because of its effectiveness in attaining linear dimension reduction. It may be used on its own or as a starting point for further study into various different dimensionality reduction approaches. Data can be altered by remapping onto a new set of orthogonal axes using a process known as projection-based principal component analysis. Following remote sensing of land resources, the pictures were classified using a support vector machine. Euroset satellite images are used to assess the suggested approach. Accuracy and kappa have both increased. It was accurate and within 95.83 % of the planned figures. The classification findings' kappa value and reasoning time were 95.87 % and 128 milliseconds, respectively. Both the model's performance and the classification effect are excellent.

## 1. Introduction

Ground information can be obtained using remote sensing technology by using various working platforms to detect remote sensing images and then process the data. This technique is known as “ground truthing.” As remote sensing technology advances, so will the visual data it generates. Image classification using remote sensing is a hot topic. Image interpretation has traditionally relied heavily on artificial visual approaches. This is a waste of time and money that does not improve accuracy. As the new standards, computers and algorithms have supplanted manual image classification. High-resolution hyperspectral photos of the objects may reveal additional information. Hyperspectral photography is the technique of photographing the whole electromagnetic spectrum, from visible to infrared, in dozens, if not hundreds, of separate and consecutive bands. This method may be used to investigate a wide range of phenomena. This imaging technology may be used to examine a wide range of scenarios. A hyperspectral imager is one of the most useful pieces of equipment for achieving this goal. There's a chance that one of these stripes may provide information about the relevant symbol. This complete photograph was most likely taken by a satellite or an aeroplane flying overhead. The visible and infrared parts of the electromagnetic spectrum provide enormous potential for research and development. It is possible that using hyperspectral photography will benefit a wide range of businesses. Food production, military service, and mineral extraction are all examples of productive activity. For each of these uses, a way needs to be made to figure out which unique hyperspectral image a given pixel came from. The abundance of feature data complicates the classification. It is critical to classify remote sensing images of land based on specific property information. Monitoring remote sensing image data is becoming increasingly important. Land classification with remote sensing imagery has become more difficult. The following new features have been added to the model because defining and classifying individual aspects is inaccurate. The proposed method extracts nine features such as colour, texture, part, and form. Using remote sensing, we were able to precisely portray sensor data. The texture of an image may be its most revealing characteristic. The proximity of pixels in an image has a significant impact on the texture exhibited. The grey level co-occurrence matrix (GLCM) is a matrix used in the research of grey level spatial dependency. It is made up of four rows and two columns. This matrix depicts the interdependence of grayscale tones throughout a particular location. The GLCM matrix may be used to determine how frequently adjacent pixels in an image have the same value. The statistical metrics may be retrieved after the GLCM matrix analysis. Textural elements allow us to estimate the spatial distribution of grey tonal shifts within a particular region. During this part of the image processing pipeline, pixels next to each other are merged into a single pixel. The overlap between the two pixels is used to determine the image's spatial values. To learn about geography, categorise the land cover using large-scale remote sensing pictures. Monitoring of the marine environment and urban planning, environmental and humanitarian aid, search-and-rescue operations, and military surveillance [1]. Images from remote sensing are hyperspectral, high-space, and high-resolution. Because photographs include more information, they may be used in novel ways [2, 3]. Land remote sensing data is big, complex, and often updated. The objective is to extract meaningful information from remote-sensing images using a computer. This promotes land utilisation.

Remote sensing images may be classified using a pattern recognition system. This technique identifies remote sensing photographs automatically. Remote sensing, classical pattern recognition, and visual interpretation are commonly used in land resource classification studies. [4]. Errors in classification may arise because the visual interpretation takes time. Discuss traditional classification schemes. These are strategies based on distance or chance. Using high-resolution remote sensing photos, the project collects data for coastal land use planning [5, 6]. The spatial motion remote sensing image sequences may be analysed to learn about the surrounding area and moving objects. Environmental issues are rarely addressed in science. Many approaches are utilised to categorise remote sensing pictures. Regression trees and least distance are two methods that outline a method for normalising NDVI data over time. To conserve the natural integrity of riparian ecosystems while simultaneously saving and extracting water for other purposes, a more thorough knowledge of the relationships between riparian vegetation and water availability is necessary. This must be done to protect the ecological stability of riparian zones. The Normalized Difference Vegetation Index, or NDVI, is a valuable measure for determining whether there have been long-term changes in the state of vegetated regions. We used regression tree analysis to investigate long-term NDVI data from semi-arid riparian zones in Australia's Namoi watershed. This investigation's testing site was the country down beneath. In addition to analysing the weather, scientists monitor groundwater levels (including temperature and precipitation). Other essential criteria in determining NDVI values include the preceding 28 days' worth of rainfall, the interflood dry period, and groundwater levels, although the maximum temperature is the most relevant. It has been proven that the highest temperature component of the NDVI data is the most critical differentiator. More rain must fall during the spring and summer for riparian zones and tree patches to maintain comparable NDVI values. This concept is referred to as the “Normalized Difference Vegetation Index.” This is because evaporation rates increase with warmth, resulting in such a rapid drop in humidity levels. Evidence suggests that dry times between floods are critical for maintaining constant NDVI values in low rainfall locations. Lower temperatures and higher precipitation levels enhance the Normalized Difference Vegetation Index (NDVI) and, by extension, plant greenness. As a result, groundwater levels fall. Time-series data is more exact, but more costly, for classifying land-cover commodities. Object-oriented classification employing fuzzy and kart decision tree techniques outperformed maximum likelihood and unsupervised methods for categorising land information [7]. The object-oriented categorization method was used. Pattern recognition classification cannot figure out where something is and cannot change it to fit new situations.

As remote sensing and computer technology progress, innovative classification approaches, such as fuzzy theories, expert systems, and artificial neural networks (ANNs) emerge. Fuzzy theory and expert system technologies are likewise cutting-edge. Remote sensing pictures may be classified using support vector machines (SVM) and k-nearest neighbours [8]. Distance is calculated by combining spatial and spectral remote sensing data with SVM class separability. Despite its modest efficiency, this method can categorise remote sensing images. Data gathered across a wide variety of wavelengths, particularly hyperspectral data, has the potential to teach us a lot about the features of the spectrum. Informative components include the location and geography of the land cover. As a result, a number of sophisticated pixel-based classifiers based on the spectral signatures of the classes have been developed over time, as have other models, such as neural networks and support vector machines. They do not, however, make use of the geographical information included in the image. As a result, the themed maps that are produced may appear congested (salt and pepper classification noise). Other solutions, such as the Markov random field and Monte Carlo optimization, have been presented (MRF). Immediately before this, the biggest disadvantage of using this technique is the amount of time required to compute.

Despite the rising complexity of today's information, even relatively tiny data sets may be fully utilised. Research is being conducted to enhance spectral and spatial light algorithms. Land cover may be correctly recognised using a terrain segmentation approach based on convolutional neural networks [9]. This method was used to partition the property. This method splits the property. To correctly categorise complex remote sensing pictures, one must keep their database knowledge up-to-date and participate in continuing training. Picture semantic segmentation using a dense coordinate transformation network may aid in the prevention of spatial data loss in remote sensing image classification [10]. This, according to experts, is a problem. This was done to remedy the problem. This method is very reliant on training data. A multiscale feature integration network with improvement phases can increase the accuracy of land remote sensing image categorization [11]. One potential advantage of multiscale feature fusion is that it may improve the semantic feature expression of multiscale targets and extremely tiny objects. To increase the network's performance, future target recognition research will almost certainly incorporate an attention mechanism. This would allow the model to collect feature-related data more effectively and efficiently, resulting in greater identification rates. If you did this, the model's ability to learn new things and find targets more accurately would both get a lot better. The classification process may be enhanced since each scale feature layer is sampled differently.

Even if a classification system can handle massive amounts of data and complex calculations, these issues persist. The algorithm's classification accuracy is poor with high-spectrum remote sensing camera images, and its efficiency and speed are nearly impossible to achieve [12]. Using ecological remote sensing photos, this research determines land resource utilisation. The following are the study's principal findings: Depth picture features are sequenced by a convolutional neural network (CNN). Remote sensing photographs may be used to derive three high-level attributes. These characteristics enable reliable classifications across a wide range of facts. When classifying pictures obtained from remote sensing, spectral, spatial, radiometric, and temporal resolutions are all taken into consideration. The bandwidth of a sensor and the sampling rate at which it collects data about its surroundings are the two primary factors that determine its spectral resolution. In addition to its other characteristics, high-quality spectral resolution may be identified by its narrow bandwidth (e.g., 10 nm). When we talk about a scene, we refer to a scene's “spatial resolution,” which refers to the capacity to discern minute distinctions between the many items in the scene (resolved). It is possible to speak of a sensor as having high radiometric resolution if it possesses the ability to capture a wide dynamic range of signals operating at varying intensities. The ability of a sensor to accomplish this task is referred to as its resolution. When the dynamic range of the image sensor is increased, the resulting photograph will have a greater number of the environment's features preserved in it. Ikonos-2's radiometric resolution lets it measure 256 different shades of grey in the energy that is reflected, while Landsat 7's sensor can only take pictures with an 8-bit depth, which is 2048 grey values. Deep learning with an SVM-based remote sensing image classifier could improve the performance of the classifier. As a result, the following subheadings are included: Section 2 describes the related research. The methodology and data collection approaches are covered in Section 3 of the research.  Section 4 will summarise the analysis, and Section 5 will present the paper's conclusion.

## 2. Related Research

Both supervised and unstructured algorithms are used in remote sensing image categorization. These methods are used in nonartificial classifications. Random forests are another popular option. It describes a technique for classifying stochastic featurespace indexes. Image categorization accuracy can be improved, but the performance with complex backdrops requires improvement. ML was used in reference to supervise and classify satellite images of national forest land use over three time periods. This strategy resulted in precise classifications. Multisensor data, according to the company, can help with semi-arid terrain classification. To assess the feasibility and value of using Sentinel-1A data's extracted backscatter intensity, texture, coherence, and colour features for urban land cover classification and to compare different multisensor land cover mapping techniques for improving classification accuracy, different permutations of the following were considered: Strength, consistency, smoothness, and colour are some of the properties that distinguish backscatter. A high-accuracy wavelet transform-based multispectral image categorization method has been developed. In multidata fusion with complex backgrounds, an RF-based classifier was used to classify land photos. Additional algorithm parameter settings are required for real-world applications.

Traditional approaches are incapable of leveraging the increased information provided by remote sensing photos. Deep learning can now categorise remote sensing photos using more high-resolution data and advances in computer technology. Deep learning is explained by CNN, DBN, and AE models. According to the reference, CNN's classification algorithm outperformed SVM without deep learning and discusses a depth learning-based remote sensing image segmentation solution. By building on shallow output, deep learning can improve image categorization accuracy over time. Shallow learning can produce a wide range of categorised outcomes. Merging network scale and node scale information is required to extract two-dimensional HSI features with varying degrees of resolution. Hyperspectral data may only consist of a small number of pixels, yet every one of them is filled with information about multiple wavelengths. Based on these findings, it was proposed to use a 2D spectrum as part of the solution. This method takes advantage of CNN's input data to create a two-dimensional spectral picture. The accuracy of the classification is enhanced since the convolution network may exploit the spatial relationships between the various spectral values. Each layer of this network is designed to alternate between maximal pooling and multiple convolutions at certain intervals. By adding BN layers between the standard 1-, 4-, and 7-layer networks, you can have more control over how data is spread and train the network faster. It can be difficult to strike the right balance between the dominant and individual visual elements. When there are few optional training examples available, CNN image segmentation is recommended [13–17]. The model, however, shows poor adaptability to image categorization using rules and scales not included in the training data. Although work based on the CNN approach has aided in the classification of remote sensing photographs, ecological resources are only occasionally considered. The result is a deep learning-based land classification using remote sensing images. This technique improves classification efficiency and accuracy while using fewer resources.

## 3. Methodology

Radiometric calibration begins with the processing of multispectral data. The grey value of the Euro Set remote sensing image is converted to the sensor's pupil radiance using ENVI for radiometric calibration [18].  Figure 1 was created in 2020 using a 2-meter panchromatic telescope and an 8-meter multispectral telescope. It is an image from a satellite.

ENVI can choose radiation calibration coefficients for the Euro Set remote sensing photos acquired over time automatically. Considering the surroundings and electromagnetic waves passing through the atmosphere to reduce atmospheric distortions, remote sensing photos must be processed. When a sensor is plugged into the software, data such as sensor height, centre point longitude and latitude, sensor type, pixel size, and imaging duration may be captured immediately. Surface reflectance images are produced by varying the imaging height, atmospheric model, and aerosol type. These images are captured by imaging equipment. The third step returns the image to its original state. Using the RPB file included with the GIF-1 image, the surface reflectance image must be “orthorectified.” This is an RPC file. The ZY-3 DEM, with an 8-meter resolution, was used to radiometrically calibrate Envi's panchromatic image and then correct it for atmospheric effects. Orthorectify the panchromatic image after radiometric calibration. Even though the ZY-3 DEM had its pixel size increased to 0.8 metres before it was fixed, it is still used.

### 3.1. Multitasking Ability

Pixel-level fusion retrieves edge and texture information for image analysis and processing. By revealing the target, you can determine whether it was correctly identified and retrieved. This indicates whether the target has been revealed. This technique preserves more information in the source image as well as the substance and details of the merged image. Fusion at the pixel level [19–21] has numerous advantages. Pixel-level picture fusion has drawbacks because it focuses on pixel operations. The computer's processing time is slow because an image has many pixels. Problems with image registration obscure the target and the composite image, resulting in inaccuracy. Image registration is widely employed in research and technology, in addition to its apparent relevance in medical and other sectors that rely on imaging technology. All imaging applications that compare people, imaging modalities, or time require this quality since it allows for the geometric alignment of datasets. Image registration seeks to create an automatic correspondence between photos by analysing several images of the same item or body part. This is accomplished through the use of several image analyses. Image registration is also known as photo fusion. Typically, the software is used to accomplish image alignment. A picture like this could have been taken at a different time or from a different angle than the photographer thought, or it could have completely hidden details that were only partly visible when the picture was taken. Before performing feature-level image fusion, the features of the source image must be extracted. A researcher examines an image of cars and people to extract feature information that can be used to identify the target. When compared to using the original image, using feature fusion for target recognition and extraction improves accuracy. Image data is compressed using feature-level fusion for computer analysis and processing. Memory and time consumption are being reduced compared to pixel-by-pixel fusion, and the merged image can be produced faster. Human cognition is required for image fusion at the decision level [22–24]. When combined with specific criteria and probabilities, this strategy can be used to determine whether additional investigation is warranted if the situation is unique and necessitates a tailored approach. The fusing process is depicted in Figure 2. The category selection could be based on information that is better suited to separate features. Deep Belief Networks (DBNs) are the outcome of unsupervised learning and combine the greatest characteristics of RBMs and belief networks (BNs). Deep belief networks (DBNs), also called multilayer belief networks (MLBNs), are a type of neural network that is fundamentally different from both perceptrons and backpropagation neural networks.

### 3.2. Categorization Scheme

DBN is subjected to learning [25], resulting in an input-label joint distribution. The RBM with many layers and the top Softmax classifiers are the structural components of the DBN model. Deep Belief Networks (DBNs) are the outcome of unsupervised learning and combine the greatest characteristics of RBMs and belief networks (BNs). Deep belief networks (DBNs), also called multilayer belief networks (MLBNs), are a type of neural network that is fundamentally different from both perceptrons and backpropagation neural networks. The precise DBN model is required to recover various types of terrain from remote sensing photographs. A well-designed DBN model can improve classification accuracy. RBM network layers can be built in the same way. The 124-250-250–2 DBN model is built based on the model's ability to classify and train.  Figure 3 depicts the model's structure.

Serial and parallel fusion techniques, covariance matrix approaches, and multi-feature histograms are used to integrate all characteristics. Then there are the characteristics. The ideal feature vector for classification is identified using evolutionary algorithms, artificial neural networks, and fuzzy logic. A specific fusion algorithm employs an end-to-end approach to create a new feature vector. A “feature vector” is a pre-arranged array of numerical characteristics of an observable event. The list is referred to as a “feature vector.” It is simply a representation of the properties needed to train a machine learning model, which then delivers a forecast based on the data used to train it. People regularly utilise qualitative data as a decision-making tool. It is possible to characterise and statistically quantify photographs by transforming their contents into Picture Feature Vectors. This is conceivable since the same-named notion is utilised in this situation, allowing it. The picture feature vector might be represented by an integer, a real number, a string of decimals, or even a binary value. All of these representations are possible. To put it simply, a feature vector is a numerical representation of an image. This is one way to think about feature vectors. This is one way to think about a feature vector. This new feature vector is used in classification and recognition [26–29]. At the start of the training phase, high-resolution images captured with remote sensing equipment are placed on a CNN with layers. If a considerable amount of the image is fixed at the same time, it is more likely that the erroneous pixel will be identified in a region of the image that is coloured a muted grey, such as a roof, after taking into consideration all of the necessary factors. This is because a larger portion of the damaged component will have been mended concurrently with the rest of it. However, when we analyse a large patch with a high resolution in addition to the features discussed above, we discover that the following is true: This is bad for two reasons: first, it wastes resources that would otherwise be used to monitor for undesirable behaviour, and second, it does not make the system more robust to disruptions. Both of these issues stem from the fact that monitoring for undesired behaviour requires resources. Each of these problems makes it harder for the system to work as a whole. The fabric of spacetime is riddled with ripples here and there (the precise arrangement of some characteristics may not be known all the time, though this may not be a major concern). As you move farther away from where the first picture was taken, it becomes less important to look at all the surrounding pixels at the high quality that they already have. When we have less data on a pixel, we need fewer characteristics to categorise it than when we have more data. Search results that are as close to perfect as a person can get in terms of finding the location of the things of interest in a search. It is critical to thoroughly analyse the scenario before forming any broad judgments about it based on what you find from your study. This is because we believe that there must be several lines of reasoning that work at various degrees of granularity. So that the work can be completed in the shortest amount of time possible, this is the single most important rule to follow in the process of generating all-encompassing semantic classifications of the many types of buildings. Recent research has focused on discovering the many ways in which FCNs may be changed to produce high-resolution and granular results. Any novel method of problem resolution may be classified into one of these three groups.

The initial need is for a sample collection of multiclass remote sensing photographs as well as a sample label. At this point, it is critical to have an image class dedicated to remote sensing photographs, an image array made up of image classes, and a label array for image classes. You must have all of these goods on hand in order to proceed with this method. It is possible to create training and test sets using the information provided by remote sensing photos. The data set includes images taken using several techniques for remote sensing. The images used to build the two sets, one for training and one for testing, are picked at random from the examples supplied below. Remote sensing practise necessitates both training and assessment, which is why images are so important in the field.

The third phase will concentrate on the development of a network with seven degrees of hierarchy. The first five levels, represented by layers one through five in the diagram above, can be examined. The convolution layer, pool layer, and interpolation layer are all found in the first three levels. To identify pool layers from convolution layers, we use the notation Pool1, Pool2, and Pool5, respectively. This helps us perceive the distinctions between the two sorts of layers more clearly. The notations Conv3 and Conv4 correspond to the single convolution layer that may be found in layers three and four, respectively. The sixth and seventh-tier links are built to accommodate the FC6 and FC7 levels.  Figure 4 demonstrates the categorization of remote sensing photos of land using a CNN network comprised of separate layers. The CNN network's network structure is trained using images collected through remote sensing. A database of test images taken with a remote sensing camera is used to figure out what each neuron's output is worth.

A process exists for the recommended multifeature fusion-based DBN classification model. There were nine traits discovered. To extract texture characteristics, the grey histogram and wavelet transform are used. The colour histogram and colour moment can be used to determine the three-color attributes of an image. Each census and scale invariant feature transformation technique yields three local shape features. The investigation will investigate nine different values. Transform the data to (0–1) after reconciling the nine features. Before and after normalization, the specified normalization function is incorporated into the formula. The DBN model's output gains additional picture features by fusing nine conciliate feature vectors. Both the computing difficulty and the classification accuracy must be considered in the final DBN model. Softmax employs the same feature fusion approach as DBN to identify land remote sensing photographs. These images are used on maps.  Figure 5 depicts image categorization with DBN (as indicated).

## 4. Experiment and Analysis

The GeForce Titan X from NVIDIA was used in the experiment. The experiment was trained using two 12 GB GPU memory units and Ubuntu 16.04. The DBN model is included in Keras and TensorFlow. Install both frameworks. Overall accuracy, recall, precision, and IoU are used to assess how well the model categorises data. The percentage of correctly classified pixels is known as the overall accuracy (OA). The recall rate is the frequency with which positively detected samples are recalled. IoU contrasts the actual and simulated samples. Positive sample occurrences are referred to as positive, whereas negative sample occurrences are referred to as negative.

### 4.1. Neurons in the Buried Layer of the Brain

Classification accuracy is evaluated for different numbers of hidden layer neurons under identical experimental conditions (120, 160, 200, 240, 280, 320, and 360).  Figure 6 depicts the results.

Changing the number of hidden neurons in the DBN model's hidden layer affects the accuracy of remote sensing image categorization. With 280 buried neurons, the classification effect was at its peak. To accurately describe input data, the DBN model necessitates many neurons in the RBM's buried layer. The unique features of a signal cannot be captured with fewer neurons than is required. Overfitting can occur when there are too many hidden layer neurons in the pretraining phase. Using the graphical representation of the identification result displayed in Figure 7, it is possible to identify residential zones even when they are dispersed and irregularly distributed over the terrain. The well-balanced layout of the project's roadways and fields contributes to the project's overall recognised impact.

The kappa coefficient and classification accuracy of the suggested technique are shown in Table 1 at 0.9587 and 95.83%, respectively. These findings clearly outperform established standards. PCA improves classification accuracy while reducing the size of the traditional 7-layer CNN network architecture. According to a deep CNN-based image recognition network available [30], the author [31] uses SVM and k-nearest neighbour algorithms to identify remote sensing images. The kappa score for problematic land resource use categories is 0.8839, suggesting poor categorization. Because of the more traditional method, the categorization effect of Reference [32] was not as strong as it could have been.

## 5. Conclusion

Land cover is essential for observing the ecological environment because seasons affect landforms, most categorization systems do not produce perfect recognition. According to these statistics, the DBN model performs best in the classification. There are 280 hidden neurons in this model, a learning rate of 0.45, and 120 unsupervised forward learning units. Land types can be accurately classified using this method. Deep learning in remote sensing is justified by the findings of 97 percent OA, 87 percent F1, and 128 milliseconds of reasoning time. These results outperformed comparable prior models. Deep learning is the most popular method for examining remote sensing photos, but it is difficult to interpret. This is even though deep learning is popular. Traditional remote sensing methods have evolved. Land use categorization is correct when ecological remote sensing photographs are separated and data is obtained using a deep learning system. This is required to improve precision agriculture and make better use of land resources. Remote sensing and deep learning are used in a method for detecting land resources. Data from remote sensing is used in the seven-layer CNN model. Remote sensing pictures are classified using TReLU and three high-level visual features. Entering these characteristics into an SVM classifier completes the classification operation. The testing time was 0.95 seconds, the accuracy was 95.83, the error was 0.0631, and the kappa was 0.9587. Training took 1.8 seconds. The results outperform those of the other assessment methods. Geometric and semantic features are frequently seen in remote sensing images. Occlusions, blurring, and distortions must be studied in future research, in addition to picture semantics. GAN models can give data with remote sensing-like distributions to fulfil the deep learning model's training data demands. This would meet these specifications. Standard deep learning networks may benefit from standard remote sensing technologies, which may improve generalisation and classification accuracy [33, 34].

## Figures and Tables

**Figure 1:** Remote-sensing image.

**Figure 2:** Feature classification and fusion.

**Figure 3:** Network structure of DBN.

**Figure 4:** The proposed method.

**Figure 5:** The classification steps with DBN.

**Figure 6:** Relationship between the hidden layer and accuracy.

**Figure 7:** Land classification.

**Table 1:** Comparative analysis of the proposed method with traditional methods.

Parameters	Decision tree classification method	SVM + KNN based method	Semantic deep learning method	The proposed method
Accuracy	87.44	88.18	93.97	95.83
Overall deficiency	16.72	11.04	08.25	06.31
Kappa value	87.30	89.40	92.84	95.87

## Data Availability

The dataset used in this research is downloaded from the Kaggle website and it is available at: https://www.kaggle.com/datasets/apollo2506/eurosat-dataset. [Accessed: 18- Jun- 2022].
